The article "PARP-1 Inhibition Repressed Imbalance of Th17 and Treg Cells in Preterm Rats with Intrauterine Infection-Induced Acute Respiratory Distress Syndrome by Reducing the Expression Level of IL-6" was published in 2022. Journal: J Healthc Eng.

# PARP-1 Inhibition Repressed Imbalance of Th17 and Treg Cells in Preterm Rats with Intrauterine Infection-Induced Acute Respiratory Distress Syndrome by Reducing the Expression Level of IL-6

**DOI:** 10.1155/2022/1255674

**Published:** 2022-02-12

**Authors:** Qian Chen, Ensheng Zhang, Chun Wang, Peipei Zhang, Lei Huang

**Affiliations:** ^1^Department of Pediatrics, Shandong Provincial Maternal and Child Health Care Hospital, No 238, Jingshi Eastern Road, Jinan 250014, Shandong Province, China; ^2^Department of Pediatrics, Guangdong General Hospital, No 106, Zhongshan Two Road, Guangzhou 510080, Guangdong Province, China

## Abstract

**Background:**

Abundant reports have uncovered an imbalance of Treg and Th17 cells in pulmonary diseases. Hereon, we intend to explore the impact of PARP-1 on the imbalance of Th17/Treg and the potential mechanism in premature rats with acute respiratory distress syndrome (ARDS).

**Methods:**

Preterm ARDS infants and healthy term infants were enrolled in this investigation. To induce a rat model of ARDS, *E.coli* suspension was given to rats through two vaginal dilator-guided intramuscular injections. H&E staining was used to perform histopathological examination. Flow cytometry was employed to assess the proportion of Th17 or Treg cells accounted for CD4^+^ T cells. ELISA was applied to measure levels of IL-6, IL-17A, and IL-10 in the serum of ARDS patients. Moreover, the mRNA and protein expression levels of PARP-1, IL-6, IL-17A, and IL-10 were detected through qRT-PCR and western blotting.

**Results:**

An increased Th17/Treg ratio was observed in preterm infants and rats with ARDS. The PARP-1 expression level was raised in the lung tissues of ARDS rats, and PARP-1 downregulation alleviated *E.coli*-induced lung injury in preterm rats. Expression levels of PARP-1, IL-6, and IL-17A were raised, and the IL-10 level was reduced in the lung tissues of rats after *E.coli* treatment, which was all reversed by PARP-1 suppression. Importantly, the ratio of Th17/Treg differentiated from purified CD4^+^ T cells of the *E.coli* + PARP-1 inhibitor group was elevated by recombinant IL-6.

**Conclusion:**

PARP-1 downregulation repressed the imbalance of Th17 and Treg cells via reducing the expression level of IL-6, implying that PARP-1 may be a promising target for ARDS therapy.

## 1. Introduction

Acute respiratory distress syndrome (ARDS) is acknowledged to be a serious form of lung injury [1]. It is caused by trauma, pneumonia, sepsis, bacterial infection, and so on [2]. Protein-induced pulmonary edema, severe hypoxemia, and loss of lung compliance are typical manifestations of ARDS [3]. Epidemiological reports have noted that about 13% of children with ARDS have a history of preterm birth or a potential history of chronic lung diseases [4]. Intrauterine infections and inflammation are closely related to early preterm births, leading to systemic inflammation in the fetus [5]. Fetal inflammation is featured by the elevated level of IL-6, which is associated with fetal lung damage [6, 7]. Previous investigation has uncovered the importance of intrauterine infection and inflammation (release of IL-6, IL-1*β*, and IL-18) in premature infants with lung injury or ARDS [6, 8]. Clinically, IL-6 has been used as a biomarker to detect neonatal ARDS [9]. However, there is limited data regarding the regulatory mechanism of IL-6 in preterm infants with ARDS.

The article "PARP-1 Inhibition Repressed Imbalance of Th17 and Treg Cells in Preterm Rats with Intrauterine Infection-Induced Acute Respiratory Distress Syndrome by Reducing the Expression Level of IL-6" was published in 2022. Journal: J Healthc Eng.

It is reported that fetal alveolar neutrophils can be activated and then reactive oxygen species (ROS) are released when maternal intrauterine infection occurs [10]. Of note, ROS-induced breaking of DNA strands results in activation of polyadenosine diphosphate ribose polymerase-1 (PARP-1), and excessive activation of PARP-1 causes cell death [11]. PARP-1 exists in all eukaryotic cells except yeast, and it is mainly involved in the modification of post-translational proteins [12]. The PAR chain on PARP-1 provides a structure (PIAS*γ*-sumoylates IKK*γ*) that leads to NF-*κ*B activation and secretion of downstream cytokines (IL-6 and TNF-*α*) [13]. A recent study has shown that activated PARP-1 upregulates the expression level of IL-6 in LPS-induced acute lung injury, which promotes the differentiation of T helper 17 (Th17) cells and represses the differentiation of CD4^+^CD25^+^Foxp3^+^ regulatory T (Treg) cells [14, 15]. IL-6 together with TGF-*β* contributes to Th17 differentiation in naive T cells and IL-6 suppresses TGF-*β*-induced Treg differentiation, thereby causing the imbalance of Treg/Th17 [16]. More importantly, the imbalance of Treg/Th17 has been demonstrated to make an impact on early ARDS [17]. The increase of Treg cells has been identified as a risk factor for ARDS patients [18, 19].

As described in prior literature, Treg cells differentiated by CD4^+^ T cells exert their functions mainly via secreting IL-10, and these cytokines are required for maintenance, induction, and enhancement of the Treg effect [20]. Th17 cells are also differentiated by CD4^+^ T cells, and IL-17A is the most characteristic cytokine of Th17 cells and mediates local tissue damage and infiltration [21].

In this study, we sought to probe the role of the PARP-1-IL-6 axis in preterm rats with intrauterine infection-induced ARDS, which will offer a promising target to ARDS treatment of premature infants.

## 2. Materials and Methods

### 2.1. Clinical Samples

This study has asked permission from the Ethical Committee of the Shandong Provincial Maternal and Child Health Care Hospital. Before enrollment, written informed consent was obtained from the guardians of all participants. From August 2018 to September 2020, 20 premature infants (birth weights <2500 g) with intrauterine infection-induced ARDS and 20 healthy term infants (normal) were enrolled in our research. The inclusion of ARDS patients complied with the Berlin definition [22]. Moreover, patients with agranulocytosis, immune-related lung diseases, or allergic alveolitis were excluded. Peripheral whole blood from the abovementioned participants was collected and then stored at −80°C until use.

The article "PARP-1 Inhibition Repressed Imbalance of Th17 and Treg Cells in Preterm Rats with Intrauterine Infection-Induced Acute Respiratory Distress Syndrome by Reducing the Expression Level of IL-6" was published in 2022. Journal: J Healthc Eng.

### 2.2. A Rat Model of *E.coli*-Induced ARDS

The pregnant Sprague–Dawley rats (age, 8–11 weeks) were bought from Slake Experimental Animal Co., Ltd. (Shanghai, China). The PARP-1 inhibitor (nicotinamide; 0.8 mmol/kg) and IL-6 (10 ng/mL) were all bought from Sigma (St. Louis, MO, USA). To induce the ARDS model, rats at embryonic day 15 (E15) were first anesthetized through intraperitoneal injection of sodium pentobarbital (2%, 40 mg/kg body weight), and then were given *E.coli* suspension (0.2 mL; Sigma) via two vaginal dilator-guided intramuscular injections on both the left and right sides of the cervix. Meanwhile, mice given saline (0.2 mL) in the same manner were regarded as controls. Specific groups of rats (*n* = 6/group) were as follows: the control group (rats received an injection of saline), the *E.coli* group (rats received an injection of *E.coli* suspension), and the *E.coli* + PARP-1 inhibitor group (before 1 h of *E.coli* injection, rats were given an intrauterine injection of 100 mg/kg PARP-1 inhibitor). Subsequently, pregnant rats (*n* = 3) of each group were anesthetized via sodium pentobarbital (40 mg/kg), and fetuses were surgically delivered on embryonic day 18 (E18). To detect successful intrauterine infection, placentae and uterine wall tissues of maternal rats were collected. In the meantime, fetal rats on E18 as well as neonatal rats on postnatal day 1 (P1) were sacrificed by cervical dislocation, and their lungs and peripheral blood were collected. The procedures regarding rats were conducted with the approval of the Laboratory Animal Welfare and Ethics Committee of Shandong Provincial Maternal and Child Health Care Hospital.

### 2.3. Isolation of CD4+ T Cells

For the peripheral blood of patients, peripheral blood mononuclear cells (PBMCs) were obtained through the standard Ficoll-Hypaque density gradient method. To obtain mononuclear cells from the lung tissues of rats, lung tissues were processed through a gentle MACS tissue dissociator (Miltenyi Biotec, Bergisch Gladbach, Germany), followed by enzymatic digestion and centrifugation. Next, CD4+ T cells were isolated from mononuclear cells according to instructions of magnetic-activated cell sorting (Stem Cell Technologies, New York, NY, USA). Then, a flow cytometer was employed to assess CD4^+^ T cells.

The article "PARP-1 Inhibition Repressed Imbalance of Th17 and Treg Cells in Preterm Rats with Intrauterine Infection-Induced Acute Respiratory Distress Syndrome by Reducing the Expression Level of IL-6" was published in 2022. Journal: J Healthc Eng.

Extracted CD4+ T cells from the lung tissues of rats in the *E.coli* + PARP-1 inhibitor group were cultured in a supernatant of bronchoalveolar lavage fluid (BALF) of the *E.coli* + PARP-1 inhibitor group, and then recombinant IL-6 (10 ng/mL) was added to incubate for 96 h.

### 2.4. Analysis of Th17 and Treg Cells via Flow Cytometry

For evaluation of Th17 cells, the surface marker antibodies against CD4 and CD25 were applied to stain CD4^+^ T cells. After treating with fixation/permeabilization buffer, CD4^+^ T cells were stained through an antibody against IL-17A. For evaluation of Treg cells, antibodies against CD4 and CD25 were employed to stain CD4^+^ T cells. Subsequently, stained cells were fixed, permeabilized, and stained with the antibody against Foxp3. In all staining procedures, isotype controls were implemented to ensure the specificity of the antibody. Ultimately, a FACSCalibur flow cytometer (BD Biosciences, San Jose, CA, USA) was employed to perform flow cytometric analysis.

### 2.5. Oxygenation Index (OI) Thresholds of Neonatal ARDS Rats

After rats were anesthetized, tracheal intubations were conducted. Pure oxygen at 7 mL/kg (120 breaths/min) was used for mechanical ventilation of rats for 20 min. Subsequently, a GEM Premier 3000 gas analyzer (Instrumentation Laboratory, Milan, Italy) was employed to measure arterial blood collected from the carotid artery. Besides, ARDS was classified as follows: OI thresholds of mild ARDS ranging from 4.0 to 7.9; OI thresholds of moderate ARDS ranging from 8.0 to 15.9; and OI thresholds of severe ARDS over 16.0 [23].

### 2.6. Enzyme-Linked Immunosorbent Assay (ELISA)

Corresponding human ELISA kits (R&D, Minneapolis, Minnesota, USA) were employed to measure serum levels of IL-6, IL-17A, and IL-10. Then, a microplate reader was used to obtain all the spectrophotometric measurements.

### 2.7. Hematoxylin-Eosin (H &E) Staining

The right lung lobes (*n* = 3/group) were fixed via 4% paraformaldehyde and embedded in paraffin, which was then cut into sagittal sections (5 *μ*m). Following deparaffinization and dehydration, these sections were stained based on the instructions of an H &E staining kit (Beyotime, Shanghai, China). Subsequently, stained samples were observed using optical microscopy.

### 2.8. The Wet/Dry Ratio of Lungs

In order to assess the wet/dry ratio (a parameter of tissue edema), harvested left lungs (*n* = 3/group) were weighed (wet weight), followed by drying in an oven at 60°C. After the lungs were dried, they were weighed (drying weight), and the wet/dry ratio was calculated based on values of the wet weight/the drying weight.

The article "PARP-1 Inhibition Repressed Imbalance of Th17 and Treg Cells in Preterm Rats with Intrauterine Infection-Induced Acute Respiratory Distress Syndrome by Reducing the Expression Level of IL-6" was published in 2022. Journal: J Healthc Eng.

### 2.9. Leukocyte and Neutrophil Counts in BALF

Rat BALF was obtained from the lavage of the right lungs. After BALF was centrifuged, the supernatant was collected for other analysis, and lysis buffer of red blood cells (Yeasen, Shanghai, China) was supplemented to remaining pellets for removing red blood cells. Then, Wright–Giemsa staining was conducted to stain the remaining BALF cells. Leukocytes were counted using optical microscopy, and neutrophils were counted according to standard morphological criteria.

### 2.10. Quantitative Real-Time PCR (qRT-PCR)

TRIzol reagent (Invitrogen, Austin, TX, USA) was applied to extract total RNA from the lung tissues of pregnant rats and newborn rats, and cDNA synthesis was performed based on a RevertAid First Strand cDNA Synthesis Kit (Thermo Fisher Scientific, San Diego, CA, USA). Then, cDNA was utilized for PCR amplification, and sequences of primers (Sangon Biotech, Shanghai, China) are displayed in Table 1. Relative expression levels of PARP-1, IL-6, IL-17A, and IL-10 normalized to GAPDH were calculated through the 2^−ΔΔCt^ method.

### 2.11. Western Blot Analysis

For obtaining total proteins, the lung tissues of rats were exposed to RIPA lysis buffer (Beyotime) and protein concentrations were measured through a BCA protein assay kit (Beyotime). Next, proteins were separated by 10% SDS-PAGE gels, followed by transfer to PVDF membranes (Millipore, Bedford, MA, USA). After being blocked with BSA (Yeasen), the primary antibodies, including PARP-1 (1 : 5000, Abcam, Cambridge, MA, USA), IL-6 (1 : 1000, Abcam), IL-17A (1 : 1000, Abcam), IL-10 (1 : 5000, Abcam), and *β*-actin (1 : 1000, Abcam), were supplemented to the membranes to incubate at 4°C overnight. Following washing with TBST, the membranes were maintained with the anti-rabbit secondary antibody (1 : 2000, Abcam). After incubation for 1 h, chemiluminescence reagents (Thermo Fisher Scientific) were used for visualization of immunoreactive bands, and Image J software (NIH, USA) was employed to analyze the intensity of those bands.

### 2.12. Statistical Analysis

Data from three replicates were presented as mean ± standard deviation, and data analysis was carried out using the GraphPad Prism 5.0 (GraphPad, USA). Moreover, the results between the two groups were compared using Student's *t*-test, and the results among multiple groups were compared via one-way ANOVA. *P* < 0.05 represented statistical significance.

The article "PARP-1 Inhibition Repressed Imbalance of Th17 and Treg Cells in Preterm Rats with Intrauterine Infection-Induced Acute Respiratory Distress Syndrome by Reducing the Expression Level of IL-6" was published in 2022. Journal: J Healthc Eng.

## 3. Results

### 3.1. The Th17/Treg Imbalance Occurs in Premature ARDS Infants

Firstly, whether an imbalance of Th17 and Treg cells occurred in premature infants of ARDS was explored. Data from flow cytometry indicated that the Th17/Treg ratio was elevated in PBMCs of ARDS infants relative to those of healthy controls (*P* < 0.001; Figure 1(a)). There existed a positive correlation between the OI thresholds of ARDS infants and the Th17/Treg ratio (*r* = 0.8253, *P* < 0.0001; Figure 1(b)). Afterward, Th17/Treg secretory cytokines were measured via ELISA, which showed that serum levels of IL-17A (*P* < 0.001) in Th17 cells and IL-10 (*P* < 0.05) in Treg cells were all boosted in ARDS infants compared to healthy controls (*P* < 0.001; Figure 1(c)). Moreover, we validated whether IL-6 was implicated in ARDS. We found that the IL-6 level in the serum of ARDS infants was elevated in comparison with healthy controls (*P* < 0.001), and it was positively associated with the Th17/Treg ratio (*r* = 0.5655, *P*=0.0094; Figure 1(d)). Shortly, the abovementioned results implied that ARDS infants presented an imbalance of Th17/Treg, and IL-6 was related to ARDS pathology.

### 3.2. PARP-1 Inhibition Alleviates Lung Injury in Rats of *E.coli*-Induced ARDS

To explore whether PARP-1 was implicated in an imbalance of Th17/Treg cells in ARDS, the role of PARP-1 was probed in the *E.coli*-induced ARDS model of rats. It was found that the placenta and uterine wall of pregnant rats (E18) showed increased infiltration of inflammatory cells after *E.coli* treatment, and the addition of PARP-1 inhibitor (nicotinamide) evidently reduced infiltration of inflammatory cells in the placenta and uterine wall of pregnant rats (E18) treated by *E.coli* (Figure 2(a)). Moreover, obvious lung infiltration, decreased lung bubble structure, and decreased alveolar number, as well as increased alveolar septum, were observed in the lung tissues of pregnant rats (E18) and neonatal rats (P1) after *E*.*coli* treatment, which was all alleviated by the addition of PARP-1 inhibitor (Figure 2(b)). During *E.coli*-triggered ARDS, the wet/dry ratio of the lungs along with the number of white blood cells and neutrophilic granulocytes in the BALF were all boosted (*P* < 0.001), followed by an evident decrease after PARP-1 inhibition in pregnant rats (E18) and neonatal rats (P1) (*P* < 0.01; Figure 2(c)). Afterward, expression levels of PARP-1, IL-17A, IL-10, and IL-6 were determined by qRT-PCR and western blot. It turned out that mRNA and protein levels of PARP-1, IL-6, and IL-17A in the lung tissues of rats were raised and the IL-10 level was reduced in response to *E.coli* treatment (*P* < 0.01), which was partially reversed by PARP-1 suppression in the lung tissues of *E.coli*-induced pregnant rats (E18) and neonatal rats (P1) (*P* < 0.05; Figures 2(d) and 2(e)). Therefore, we inferred that PARP-1 downregulation alleviated lung injury in *E*.*coli*-induced rats.

The article "PARP-1 Inhibition Repressed Imbalance of Th17 and Treg Cells in Preterm Rats with Intrauterine Infection-Induced Acute Respiratory Distress Syndrome by Reducing the Expression Level of IL-6" was published in 2022. Journal: J Healthc Eng.

### 3.3. PARP-1 Downregulation Reduces Imbalance of the Th17/Treg Ratio in *E*.*coli*-Induced Newborn Rats

After that, we determined whether PARP-1 made an impact on the imbalance of the Th17/Treg in rats. As shown in Figure 3(a), the ratio of Th17/Treg in the lung tissues of E18 rats and P1 rats was raised in response to *E.coli* treatment (*P* < 0.001), and the addition of PARP-1 inhibitor led to a reduction of the Th17/Treg ratio (*P* < 0.01 or *P* < 0.001). Then, the impact of the PARP-1 inhibitor on rat OI thresholds was assessed. It turned out that *E.coli* treatment resulted in the increase of OI thresholds (*P* < 0.0001), which was reversed by PARP-1 suppression in P1 rats (*P* < 0.01; Figure 3(b)). Accordingly, the correlation between the Th17/Treg ratio and the OI thresholds of P1 rats was analyzed in different treatments. As shown in Figure 3(c), the Th17/Treg ratio and OI thresholds exhibited a positive correlation in P1 rats with *E.coli* treatment (*r* = 0.8563, *P* < 0.0001). Our data illustrated that the imbalance of Th17 and Treg cells was repressed by PARP-1 inhibition, and it was positively correlated with OI thresholds in *E.coli*-induced P1 rats.

### 3.4. Increased IL-6 Promotes Th17/Treg Imbalance in the Lung Tissues of Rats Induced by *E*.*coli* and PARP-1 Inhibitor

Another issue we verified was whether IL-6 participated in the impact of the PARP-1 inhibitor on Th17/Treg imbalance. According to data of flow cytometry analysis, we found that the ratio of Th17 and Treg cells differentiated from purified CD4+ T cells in the lung tissues of rats induced by *E.coli* and PARP-1 inhibitor was raised by recombinant IL-6 (*P* < 0.05; Figure 4).

## 4. Discussion

In the past few years, great progress has been made in the exploration of ARDS pathology [24, 25], and ARDS is reported to be strongly associated with the inordinate immune response of the lungs [26, 27]. Importantly, a recent study has demonstrated that a differentiation imbalance of Th17 and Treg cells occurs in ARDS and is responsible for ARDS development [17]. In line with the abovementioned findings, we discovered that the Th17/Treg ratio was elevated in PBMCs of premature ARDS infants compared to healthy controls and that it was positively correlated with the OI thresholds of premature ARDS infants. These results indicated that the imbalance of Th17 and Treg cells contributed to ARDS development. At the same time, inflammatory factors secreted by Th17 and Treg cells were measured using ELISA, which showed that serum levels of both IL-17A in Th17 cells and IL-10 in Treg cells were raised in premature infants with ARDS. Furthermore, given the significance of IL-6 in the clinical diagnosis of ARDS patients [9], its protein level was determined. It turned out that the protein level of IL-6 was boosted in the serum of premature ARDS infants relative to that of healthy controls, and it was positively associated with the Th17/Treg ratio.

The article "PARP-1 Inhibition Repressed Imbalance of Th17 and Treg Cells in Preterm Rats with Intrauterine Infection-Induced Acute Respiratory Distress Syndrome by Reducing the Expression Level of IL-6" was published in 2022. Journal: J Healthc Eng.

Previously, convincing evidence has highlighted that PARP-1 exerts a critical role in lung-related diseases, such as asthma, silicosis, and ARDS [28]. PARP-1 downregulation has been reported to suppress inflammation in a mouse model of asthma [29]. Here, we demonstrated that PARP-1 downregulation repressed inflammation through reducing the infiltration of inflammatory cells in *E.coli*-induced rats, which was similar to prior work. Moreover, we discovered that the wet/dry ratio of the lungs as well as the number of white blood cells and neutrophilic granulocytes in BALF were reduced after PARP-1 inhibition in *E*.*coli*-induced rats, showing a protective role of the PARP-1 inhibitor against lung injury in ARDS.

Since the imbalance of Th17/Treg is important for ARDS development based on our findings, we then probed the impact of PARP-1 inhibitor on the imbalance of Th17/Treg. It was found that the addition of the PARP-1 inhibitor reduced the *E*.*coli*-mediated increase of the Th17/Treg ratio in lung tissues in rats. Meanwhile, the increased level of IL-17A and the decreased level of IL-10 were observed in the lung tissues of rats after *E*.*coli* treatment, which was all reversed by PARP-1 suppression. Taken conjointly, these results indicated that PARP-1 downregulation repressed the imbalance of Th17/Treg in ARDS. And our findings were similar to previous reports where PARP-1 up-regulation was found to promote differentiation of Th17 cells and suppress differentiation of Treg cells in LPS-induced lung injury [14, 15]. Our data highlighted the potential of the PARP-1 inhibitor as a treatment for ARDS.

Emerging evidence has manifested that IL-6 can facilitate Th17 differentiation and suppress Treg differentiation in naive T cells, causing the imbalance of Treg and Th17 cells [16]. More importantly, PARP-1 activation is uncovered to promote the expression level of IL-6 in LPS-induced acute lung injury, which promotes the differentiation of Th17 cells and reduces the differentiation of Treg cells [14, 15]. Therefore, when delving into underlying mechanisms associated with the role of PARP-1 in ARDS, whether IL-6 was regulated by PARP-1 and whether IL-6 could reverse the impact of PARP-1 on the imbalance of Th17/Treg were verified in *E*.*coli*-induced rats. Similarly, we explicitly found that the mRNA and protein level of IL-6 were reduced by the PARP-1 inhibitor in the lung tissues of *E.coli*-induced pregnant rats and neonatal rats. In the meantime, we observed that the ratio of Th17/Treg was raised by IL-6 addition in the lung tissues of rats induced by *E.coli* and PARP-1 inhibitor. Combining these findings, we inferred that PARP-1 regulated the imbalance of Th17/Treg by affecting the IL-6 expression level in *E*.*coli*-induced rats. These results suggested that the PARP-1-IL-6 pathway may be a new mechanism to regulate the imbalance of Th17/Treg, which is pivotal for alleviating ARDS pathogenesis.

The article "PARP-1 Inhibition Repressed Imbalance of Th17 and Treg Cells in Preterm Rats with Intrauterine Infection-Induced Acute Respiratory Distress Syndrome by Reducing the Expression Level of IL-6" was published in 2022. Journal: J Healthc Eng.

To conclude, we demonstrated that PARP-1 downregulation repressed the imbalance of Th17 and Treg cells, and it alleviated lung injury in the *E.coli*-induced rat model of ARDS. Besides, our data provided a novel mechanism for ARDS, which indicated that PARP-1 inhibition impaired the imbalance of Th17 and Treg cells by reducing the expression level of IL-6 in *E*.*coli*-induced rats.

## Figures and Tables

**Figure 1:** The Th17/Treg imbalance occurs in premature ARDS infants. (a) Flow cytometric analysis was performed to assess the proportion of Th17 cells and Treg cells in CD4^+^ cells from PBMCs of ARDS patients and healthy controls. (b) The correlation between the Th17/Treg ratio and OI thresholds in ARDS patients and healthy controls was analyzed using Spearman's method. (c) ELISA was applied to measure serum levels of IL-17A and IL-10 in ARDS patients and healthy controls. (d) ELISA was used to determine the relative serum level of IL-6 in ARDS patients and healthy controls, and the correlation between the Th17/Treg ratio and the relative serum level of IL-6 in ARDS patients and healthy controls was analyzed using Spearman's method. ^*∗*^*P* < 0.05, ^*∗∗*^*P* < 0.01, ^*∗∗∗*^*P* < 0.001, Vs. normal. Each experiment was repeated three times.

**Figure 2:** PARP-1 inhibition alleviates lung injury in rats with *E.coli*-induced ARDS. (a) HE staining was used to perform the histopathological examination of the placenta and uterine wall in rats. (b) HE staining was used to perform the histopathological examination of lung tissues in rats. (c) The wet/dry ratio of the lungs, as well as the numbers of white blood cells and neutrophils, was determined in rats. (d–e) qRT-PCR and western blot were performed to determine the mRNA and protein expression levels of PARP-1, IL-6, IL-17A, and IL-10 in the lung tissues of rats. ^*∗∗*^*P* < 0.01, ^*∗∗∗*^*P* < 0.001, ^*∗∗∗∗*^*P* < 0.0001, Vs. control. ^#^*P* < 0.05, ^##^*P* < 0.01, ^###^*P* < 0.001, Vs. *E.coli*. Each experiment was repeated three times.

The article "PARP-1 Inhibition Repressed Imbalance of Th17 and Treg Cells in Preterm Rats with Intrauterine Infection-Induced Acute Respiratory Distress Syndrome by Reducing the Expression Level of IL-6" was published in 2022. Journal: J Healthc Eng.

**Figure 3:** PARP-1 downregulation reduces the imbalance of the Th17/Treg ratio in CD4^+^ T cells from *E.coli*-induced newborn rats. (a) Flow cytometric analysis was performed to assess the proportion of Th17 cells and Treg cells in CD4^+^ cells from the lung tissues of rats. (b) Oxygenation index (OI) thresholds were assessed in rats. (c) The correlation between the Th17/Treg ratio and OI thresholds in rats was analyzed using Spearman's method. ^*∗∗∗*^*P* < 0.001, ^*∗∗∗∗*^*P* < 0.0001, Vs. control. ^##^*P* < 0.01, ^###^*P* < 0.001, Vs. *E*.*coli*. Each experiment was repeated three times.

**Figure 4:** Increased IL-6 promotes Th17/Treg imbalance in PARP-1 inhibitor and *E.coli* cotreated CD4^+^ T cells from lung tissues of rats. Flow cytometric analysis was performed to assess the proportion of Th17 cells and Treg cells in CD4^+^ cells from the lung tissues of rats in the *E*.*coli* + PARP-1 inhibitor group. ^*∗*^*P* < 0.05, ^*∗∗*^*P* < 0.01, Vs. *E*.*coli* + PARP-1 inhibitor. Each experiment was repeated three times.

**Table 1:** The primer sequences for qRT-PCR in this study.

Genes		Sequences (5'∼3')
PARP-1	Forward	GAGTGGGCACAGTTATCGGC
	Reverse	CCAGGCATTTCCAGTCTTCTCT
IL-6	Forward	CAACGATGATGCACTTGCAGA
	Reverse	CTCCAGGTAGCTATGGTACTCCAGA
IL-10	Forward	GGGGCCAGTACAGCCGGGAA
	Reverse	CTGGCTGAAGGCAGTCCGCA
IL-17A	Forward	GCAAAAGTGAGCTCCAGAAGG
	Reverse	TCTTCATTGCGGTGGAGAGTC
GAPDH	Forward	AGGTCGGTGTGAACGGATTTG
	Reverse	GGGGTCGTTGATGGCAACA

## Data Availability

All datasets for the analysis in the present study are available upon reasonable request from the corresponding author.

## Abbreviations

ARDS: Acute respiratory distress syndrome
ROS: Reactive oxygen species
PARP-1: Polyadenosine diphosphate ribose polymerase-1
Th17: T helper 17
Treg: Regulatory T
PBMCs: Peripheral blood mononuclear cells
OI: Oxygenation index
ELISA: Enzyme-linked immunosorbent assay
H&E: Hematoxylin-eosin
BALF: Bronchoalveolar lavage fluid
qRT-PCR: Quantitative real-time PCR.
